# Urine Albumin/Creatinine Ratio and Microvascular Disease in Elderly Hypertensive Patients without Comorbidities

This article has been retracted.

**DOI:** 10.1155/2021/5560135

**Published:** 2021-02-13

**Authors:** Guihua Jian, Wenjun Lin, Niansong Wang, Junnan Wu, Xianfeng Wu

**Affiliations:** ^1^Department of Nephrology, Shanghai Jiao Tong University Affiliated Sixth People's Hospital, Shanghai, China; ^2^Clinical Research Center for Chronic Kidney Disease, Shanghai Jiao Tong University Affiliated Sixth People's Hospital, Shanghai, China

## Abstract

**Objectives:**

A high urine albumin/creatinine ratio (UACR) is associated with microvascular disease in hypertensive patients. However, hypertensive patients frequently have other comorbidities. Thus, it is difficult to distinguish the role of UACR from that of comorbidities in microvascular disease. The aim of this study was to evaluate the association between UACR and microvascular disease in elderly hypertension patients without comorbidities.

**Methods:**

A cross-sectional cohort study of 2252 essential hypertension patients aged 65-94 years without comorbidities between January 1, 2016, and December 31, 2017, was conducted. Microvascular disease was evaluated by hypertension retinopathy (HR). Multivariable adjusted odds of HR by UACR quartiles were determined using logistic regression.

**Results:**

The HR prevalence was 22.1% (*n* = 472) among the cohort study and was significantly different among UACR quartiles (19.7%, 20.3%, 22.0%, and 26.4% in quartiles 1, 2, 3, and 4, respectively, *P* = 0.036). After adjustment for covariates, higher UACR (odds ratio (OR) = 1.42, 95% confidence interval (CI) 1.05-1.92, quartile 4 versus 1) were significantly associated with HR. Among male patients, higher UACR (OR = 1.65, 95% CI 1.07-2.55, quartile 4 versus 1) were significantly associated with HR after adjustment for covariates. Among female patients, however, 64% and 40% increased odds of HR were noted in the highest and lowest UACR (quartiles 4 and 1, respectively) compared to UACR quartile 2.

**Conclusions:**

Microvascular disease was associated with higher UACR in elderly male essential hypertension patients without comorbidities but was associated with lower and higher UACR in female patients without comorbidities.

## 1. Introduction

Hypertension is a growing global health problem and a significant risk factor for the development of various cardiovascular diseases, including coronary heart disease, stroke, microvascular disease (MVD), and chronic kidney disease [1–4]. MVD is considered a crucial pathway in the development and progression of cardiometabolic and renal disease and is associated with increased cardiovascular mortality [5]. In the general population, age, sex, hypertension, dyslipidemia, hyperglycemia, obesity, albuminuria, and smoking are significant determinants of MVD [6–10]. It is well known that MVD is the result of hypertension [11, 12]. Patients with hypertension often suffer from other comorbidities, such as diabetes, dyslipidemia, hyperglycemia, obesity, and proteinuria, and harmful habits such as smoking and drinking. Thus, it is difficult to distinguish the role of these risk factors from that of comorbidities in MVD.

A meta-analysis study reported that albuminuria was associated with cerebral small vessel disease, indicating shared MVD in the kidney and the brain [10]. Another study from the United Kingdom also reported that albuminuria is associated with a narrower and wider arteriolar caliber in patients aged 45-84 years without baseline clinical cardiovascular disease [13]. However, patients with diabetes or smoking were not excluded in these studies. Therefore, it is difficult to distinguish the role of albuminuria from that of comorbidities in MVD. In the present study, to reduce the effect of comorbidities and harmful habits on MVD, we included those without comorbidities and free of current smoking and drinking. Besides, an elevated urine albumin/creatinine ratio (UACR) below the proteinuria level, i.e., microalbuminuria, has long been recognized as a marker of kidney disease and increased cardiovascular risk, and MVD is a consequence of hypertension and elderly age was associated with MVD [11, 12, 14]. To reduce the effect of hypertension and elderly age on MVD, we only included elderly age patients with hypertension. Thus, we aimed to evaluate the association between UACR and MVD in elderly Chinese hypertensive patients without comorbidities.

## 2. Materials and Methods

### 2.1. Study Population

The study was a cross-sectional cohort study of 2252 men and women aged 65-94 years (mean age 71.8 years), without clinical comorbidities, recruited from the Gumei community (Minhang District, Shanghai, China) between January 1, 2016, and December 31, 2017. This study was designed to investigate the prevalence of MVD and its predictors. Elderly essential hypertension patients with symptoms or a history of medical or treatment for comorbidities were excluded. Patients with current smoking or drinking were also excluded. Patients with eGFR less than 60 mL/min/1.73 m^2^ may possibly develop vascular dysfunctions and complications [15, 16]. Thus, we also excluded those with eGFR < 60 mL/min/1.73 m^2^. No patients were involved in setting the research question or outcome measures or were involved in the design or implementation of the study. This study was conducted according to the principles expressed in the Declaration of Helsinki. The Ethics Committees of the Gumei Community Health Center approved the protocol of this cross-sectional study and waived the need for written informed consent because the data were analyzed anonymously.

### 2.2. Urine Albumin/Creatinine Ratio

The patients provided basic health information and a spot urine specimen generally immediately after arriving in the morning at the Gumei Community Health Center. Urine albumin and creatinine were measured at the Clinical Chemistry Laboratory at the Affiliated Sixth People's Hospital, Shanghai Jiao Tong University. A spot UACR in milligrams/grams was then calculated for all patients. Patients with reasons for a false-positive UACR test were excluded. Albuminuria was then defined as a UACR ≥ 30 mg/g for men and women. This definition includes both microalbuminuria (UACR ≥ 30-299 mg/g) and macroalbuminuria (UACR ≥ 300 mg/g) [13].

### 2.3. Retinal Photography

The retinal microvasculature reflects cumulative small vessel damage from hypertension and other vascular processes [12]. Thus, in the present study, MVD was evaluated by retinal photography. Retinal photography was performed using a standardized protocol [17, 18]. A 45-degree 6.3-megapixel nonmydriatic camera was used to photograph the optic discs and macula of both eyes of each subject. These photographs were sent to the Affiliated Sixth People's Hospital, Shanghai Jiao Tong University, for evaluation of retinal pathology. Trained graders were blinded to participant characteristics. The HR classification is based on Mitchell–Wong classification systems [19].

### 2.4. Covariates

All patients completed self-administered questionnaires and were interviewed and checked by trained researchers. In the morning of the participant's first arrival at the examination, fasting blood and urine samples were collected. Baseline characteristics were recorded, including age, sex, body mass index (BMI), systolic blood pressure (BP), diastolic BP, neutrophil to lymphocyte (N/L) ratio, fasting blood glucose, cholesterol, triglycerides, high-density lipoprotein cholesterol (HDL-c), low-density lipoprotein cholesterol (LDL-c), and estimated glomerular filtration rate (eGFR). Systolic BP and diastolic BP were measured three times, and the average was used as the final value after patients had been seated and resting quietly for more than five minutes with feet on the ground and back supported (OMRON Corporation, Kyoto, Japan) [20]. Hypertension was defined as a systolic BP ≥ 140 mmHg or a diastolic BP ≥ 90 mmHg. Patients currently using antihypertensive medications were also classified as positive for hypertension [21]. BMI was calculated as the weight in kilograms divided by the square of height in meters. Residual renal function was assessed by eGFR using the Chronic Kidney Disease Epidemiology Collaboration creatinine equation [22].

### 2.5. Statistical Analysis

Missing values for all variables were less than 10% in the present study. The missing data is estimated using the missForest method, which is a nonparametric method that processes different types of variables simultaneously [23]. Means ± standard deviations and percentages were used to summarize the characteristics of the study sample by UACR quartiles. Continuous and categorical variables were compared across quartiles of UACR using analysis of variance (ANOVA) and chi-square tests, respectively. We used the quartile with the lowest HR prevalence as a reference (quartiles with higher HR prevalence versus quartile with the lowest HR prevalence). Three models were created to assess potential confounding. Three different logistic regression models were examined so that changes in the parameter estimate with the addition of demographic and laboratory factors could be examined. Unadjusted associations were first examined, followed by adjustments for age and sex. Next, BMI, systolic BP, diastolic BP, N/L ratio, fasting blood glucose, cholesterol, triglycerides, HDL-c, LDL-c, and eGFR were added to examine whether the association of the UACR quartiles with HR was independent of confounding factors. Models were then repeated in the male and female patients. Statistical analyses were performed using the R package 3.6.0 (https://www.r-project.org/).

## 3. Results

### 3.1. Baseline Characteristics

Of the 2252 patients, 112 had eGFR < 60 mL/min/1.73 m^2^, leaving 2140 for this analysis. Of 2140 patients with the mean age of 71.8 ± 5.6 years, 48.8% were male. UACR ranged from 0.4 to 1123.7 mg/g in the cohort study. Patients with UACR were classified into quartiles: quartile 1 < 10.5 mg/g, quartile 2 = 10.5-19.5 mg/g, quartile 3 = 19.6-36.5 mg/g, and quartile 4 ≥ 36.6 mg/g. The characteristics of the study patients by UACR quartiles are shown in Table 1.

Patients with the highest UACR (quartile 4) had higher systolic BP, diastolic BP, fasting blood glucose, triglycerides, and HDL-c but lower eGFR compared to patients in the lower UACR quartiles 1-3.  Table 2 shows the characteristics of male and female patients by UACR quartiles.

Similar differences of characteristics among UACR quartiles were observed in male and female patients. The characteristics of the study patients by sex are shown in Table 3.

### 3.2. The HR Prevalence

Figure 1 shows the HR prevalence by UACR quartiles among the patients.

The HR prevalence was 22.1% (*n* = 472) in the cohort population. The HR prevalence was highest in quartile 4 (26.4%) and lowest in quartile 1 (19.7%). Among male patients, the HR prevalence also was highest in quartile 4 (27.5%) and lowest in quartile 1 (17.4%). However, among female patients, the HR prevalence was highest in quartile 4 (25.4%) but lowest in quartile 2 (17.4%).

### 3.3. The Association between UACR and HR

Table 4 shows the results of the logistic regression analyses for UACR quartiles.

Among the cohort study, higher UACR (quartile 4) was associated with 46% increased odds of HR compared to UACR quartile 1 in the unadjusted model (model 1). Further adjustment for demographic and laboratory factors mildly reduced the parameter estimate. In the fully adjusted model (model 3), higher UACR (quartile 4) was associated with 42% increased odds of HR compared to UACR quartile 1 (95%confidence interval (CI) 1.05-1.92).

### 3.4. The Association between UACR and HR Stratified by Sex

Albuminuria prevalence (UACR ≥ 30.0 mg/g) was not significantly different between men (30.6%) and women (31.8%), and the presence of albuminuria was not significantly associated with sex (male versus female, OR = 1.06, 95% CI 0.88-1.27). Interaction terms showed no significant modification by sex on the association between UACR and HR. However, due to the established clinical importance that sex holds for the risk of HR, we further explored the association between UACR quartiles and the presence of HR in analyses in male and female patients (Table 5).

Among male patients, similar trends were observed compared to associations noted in the cohort study with the highest UACR quartile 4 associated with an increased odd of HR compared to the lowest UACR quartile 1. Among male patients, higher UACR (quartile 4) was associated with 65% increased odds of HR compared to UACR quartile 1 (95% CI 1.07-2.55) in the fully adjusted model (model 3). However, among female patients, when using quartile 1 as a reference, we did not find the association between UACR and HR (data not shown). Nonetheless, among female participants, the HR prevalence was lowest in quartile 2 (17.4%). When using quartile 2 as a reference, higher UACR (quartile 4) was associated with 61% increased odds of HR in the unadjusted model (model 1). In the fully adjusted model (model 3), higher UACR (quartile 4) remained to be associated with 61% increased odds of HR compared to UACR quartile 2 (95% CI 1.06-2.45). Besides, 40% increased odds of HR were noted in the lowest UACR (quartile 1) compared to UACR quartile 2.

## 4. Discussion

In this study, we found that higher UACR was independently associated with an increased prevalence of HR in elderly male hypertensive patients without comorbidities. Besides, we noted a U-shaped distribution of HR prevalence across the range of UACR with the higher prevalence of HR consistently seen among female patients with higher or lower UACR. In part, this may be explained because sex differences in demographics might explain the observed differences in the prevalence of HR between men and women.

HR is thought to be microvascular damage caused by aging, hypertension, and other processes, reflecting endometrial thickening and medial hyperplasia, transparency, and sclerosis [24]. Because similar pathological features are also seen in the coronary and renal arterioles in patients with hypertension, changes in the retinal arterioles may provide useful information about the state of systemic microcirculation in health and disease [25]. In the present study, therefore, we used HR to evaluate MVD. The independent association between UACR and HR likely reflected microvascular processes in elderly hypertensive patients without comorbidities. For the first time, to minimize the effect of comorbidities and harmful habits on MVD, we excluded those with comorbidities and harmful habits. Thus, the independent associations between UACR and MVD may be more reliable and convincing than those reported by previous studies [10, 13]. A study from the United Kingdom examined the association between retinal arteriolar and venular caliber and the presence of albuminuria (micro- or macroalbuminuria) among participants aged 45-84 years without baseline clinical cardiovascular disease [13]. The authors reported that albuminuria is associated with a narrower and wider arteriolar caliber. Nonetheless, they did not exclude those with hypertension, diabetes, or harmful habits, which suggested that associations between the arteriolar caliber and the presence of incident albuminuria may be mediated by hypertension, diabetes, and harmful habits. Another study examined the association between retinal vascular diameter and chronic kidney disease in a population-based cohort of 3280 community-dwelling adults aged 40-80 years living in Singapore. The authors reported that MVD was also found to be positively associated with both eGFR and micro/macroalbuminuria [26]. Similarly, patients with diabetes, drinking, or smoking were not excluded, which may lead to under- or overestimation of the association between MVD and micro/macroalbuminuria.

To date, the association between sex and albuminuria is inconsistent in the previous studies [27, 28]. Men and Blacks have a higher UACR than do women and Whites and may thereby have an increased risk of microvascular and macrovascular disease [27]. However, another study showed that in the multivariate-adjusted model, female sex (OR = 1.62; 95% CI 1.29-2.05) was independently associated with microalbuminuria [28]. In the present study, albuminuria prevalence was not significantly different between men and women and the presence of albuminuria was not significantly associated with sex. These findings in our study may be more reliable due to excluding those with comorbidities or harmful habits, which may reduce the effect of comorbidities and harmful habits on the association between albuminuria and sex.

The prevalence, progression, and pathophysiology of both MVD and macrovascular disease are different in the two sexes [29–32]. Nonetheless, there are few studies focusing on sex-dependent differences in the association between UACR and MVD. In the present study, we found that there were sex-dependent differences in the association between UACR and MVD. Among male patients, the highest UACR (quartile 4) had a 1.65-fold risk of MVD compared to the lowest UACR (quartile 1) after adjustment for covariates. Among female patients, however, the highest and lowest UACR (quartiles 4 and 1) had 1.64- and 1.40-fold risk of MVD compared to UACR quartile 2. Therefore, among men patients, higher UACR was independently associated with an increased prevalence of MVD, but a U-shaped distribution of MVD prevalence across the range of UACR with the higher prevalence of MVD consistently was seen among female patients with higher or lower UACR.

The strength of our study was to reduce the effect of comorbidities and harmful habits on MVD, and we excluded those elderly hypertensive patients with comorbidities or harmful habits. Thus, these findings may be more reliable and convincing in our study. There are some limitations of this work to be noted. First, we did not exclude those with macroalbuminuria, which may lead to selective bias. Because the causes of macroalbuminuria may be attributed to other diseases rather than hypertension, the selective bias may under- or overestimate the prevalence of MVD. Secondary, we have not documented antihypertensive drugs, such as renin-angiotensin, which play a crucial role in the treatment of albuminuria. Finally, because this is a cross-sectional cohort, we cannot exclude the possibility of residual or unmeasured confounding. A further prospective longitudinal study should be conducted to evaluate whether the UACR management may improve the MVD process in elderly hypertensive patients.

In summary, we found that there were sex-dependent differences in the association between UACR and MVD in those elderly hypertensive patients without comorbidities. Among men patients, higher UACR was independently associated with an increased prevalence of MVD, but a U-shaped distribution of MVD prevalence across the range of UACR with the higher prevalence of MVD consistently was seen among female patients with higher or lower UACR. Thus, different UACR management should be conducted for elderly men and women hypertensive patients.

## Figures and Tables

**Figure 1:** Prevalence of hypertension retinopathy by UACR quartiles and by the presence of sex. UACR: urine albumin/creatinine ratio.

**Table 1:** Characteristics and Mitchell–Wong classification in the cohort study by quartiles of UACR.

	Quartile 1 (*n* = 534)	Quartile 2 (*n* = 538)	Quartile 3 (*n* = 533)	Quartile 4 (*n* = 535)
Age (years)	71.8 ± 5.5	71.3 ± 5.5	72.1 ± 5.7	71.9 ± 5.8
Male (%)	264 (49.4)	262 (48.7)	263 (49.3)	255 (47.7)
BMI (kg/m^2^)	21.9 ± 3.2	21.9 ± 3.1	21.9 ± 3.1	22.3 ± 3.5
Systolic BP (mmHg)	136.7 ± 17.4	139.0 ± 17.5	142.1 ± 17.6^∗^	145.8 ± 15.8^∗^
Diastolic BP (mmHg)	79.3 ± 10.6	79.2 ± 10.4	81.0 ± 11.0^∗^	81.5 ± 11.9^∗^
N/L ratio	1.77 ± 0.89	1.77 ± 0.73	1.84 ± 1.05^∗^	1.79 ± 0.92
Fasting blood glucose (mg/dL)	98.4 ± 17.0	104.6 ± 16.1^∗^	106.7 ± 19.5^∗^	110.0 ± 24.0^∗^
Cholesterol (mg/dL)	202.5 ± 37.1	206.3 ± 38.5	207.3 ± 41.8	208.8 ± 42.7^∗^
Triglycerides (mg/dL)	132.6 ± 98.9	138.9 ± 77.6	147.5 ± 85.4^∗^	147.6 ± 87.6^∗^
HDL-c (mg/dL)	61.0 ± 13.1	64.6 ± 14.7^∗^	63.6 ± 13.5^∗^	64.8 ± 14.3^∗^
LDL-c (mg/dL)	113.8 ± 30.1	112.6 ± 29.9	113.5 ± 31.2	113.0 ± 32.0
eGFR (mL/min/1.73 m^2^)	90.8 ± 20.7	87.7 ± 18.8	80.0 ± 19.0^∗^	78.5 ± 18.3^∗^
Mitchell–Wong classification				
None (%)	429 (80.3)	429 (79.7)	416 (78.0)	394 (73.6)
Mild (%)	98 (18.4)	90 (16.7)	104 (19.5)	118 (22.1)
Moderate (%)	7 (1.3)	16 (3.0)	13 (2.4)	19 (3.6)
Malignant (%)	0 (0.0)	3 (0.6)	0 (0.0)	4 (0.7)

^∗^ *P* < 0.05 compared to quartile 1. UACR: albumin/creatinine ratios; BMI: body mass index; BP: blood pressure; N/L: neutrophil to lymphocyte ratio; HDL-c: high-density lipoprotein cholesterol; LDL-c: low-density lipoprotein cholesterol; eGFR: estimated glomerular filtration rate.

**Table 2:** Characteristics and Mitchell–Wong classification in elderly male and female patients by quartiles of UACR.

	Male				Female			
	Quartile 1 (*n* = 264)	Quartile 2 (*n* = 262)	Quartile 3 (*n* = 263)	Quartile 4 (*n* = 255)	Quartile 1 (*n* = 270)	Quartile 2 (*n* = 276)	Quartile 3 (*n* = 270)	Quartile 4 (*n* = 280)
Age (years)	72.2 ± 5.7	71.2 ± 5.2	72.5 ± 5.9	72.5 ± 5.8	71.5 ± 5.4	71.4 ± 5.7	71.7 ± 5.6	71.3 ± 5.7
BMI (kg/m^2^)	21.8 ± 3.2	21.9 ± 2.9	22.0 ± 3.1	22.4 ± 3.3	22.0 ± 3.2	22.0 ± 3.2	21.9 ± 3.1	22.3 ± 3.7
Systolic BP (mmHg)	135.2 ± 16.6	139.5 ± 17.4	142.8 ± 18.0^∗^	145.1 ± 19.0^∗^	138.1 ± 18.1	138.4 ± 17.5	141.5 ± 17.2	146.4 ± 18.7^¶^
Diastolic BP (mmHg)	78.1 ± 10.2	79.3 ± 10.8	81.0 ± 10.9	81.1 ± 12.5^∗^	80.4 ± 10.8	79.1 ± 10.0	81.1 ± 11.1	82.0 ± 11.3^¶^
N/L ratio	1.72 ± 0.71	1.77 ± 0.73	1.84 ± 1.05	1.84 ± 1.16	1.82 ± 1.04	1.74 ± 0.69	1.89 ± 1.31	1.74 ± 0.63
Fasting blood glucose (mg/dL)	98.1 ± 16.6	104.8 ± 16.3^∗^	106.0 ± 17.3^∗^	110.6 ± 25.1^∗^	98.7 ± 17.4^¶^	104.4 ± 16.0	107.4 ± 21.4	109.5 ± 22.9^¶^
Cholesterol (mg/dL)	201.8 ± 39.3	206.7 ± 37.3	209.0 ± 41.5^∗^	207.8 ± 42.5	203.2 ± 34.9	205.9 ± 39.8	205.6 ± 42.0	210.0 ± 43.0
Triglycerides (mg/dL)	135.5 ± 112.9	140.4 ± 84.6	149.8 ± 90.6	148.9 ± 96.0	129.8 ± 83.0	137.4 ± 70.5	145.3 ± 80.1	146.4 ± 79.3
HDL-c (mg/dL)	60.4 ± 14.2	64.5 ± 14.5^∗^	64.2 ± 12.6^∗^	64.4 ± 14.0^∗^	61.7 ± 13.1^¶^	64.6 ± 14.9	63.0 ± 14.3	65.1 ± 14.6
LDL-c (mg/dL)	113.5 ± 32.7	120.7 ± 35.4	114.0 ± 31.4	111.9 ± 32.7	114.1 ± 27.3	111.7 ± 30.7	113.1 ± 31.1	113.9 ± 31.4
eGFR (mL/min/1.73 m^2^)	89.9 ± 19.2	86.7 ± 35.4	83.7 ± 17.4^∗^	79.5 ± 16.7^∗^	87.9 ± 18.6	89.0 ± 19.3	82.9 ± 18.7^¶^	78.4 ± 17.9^¶^
Mitchell–Wong classification								
None (%)	218 (82.6)	201 (76.7)	204 (77.6)	185 (72.5)	211 (78.1)	228 (82.6)	212 (78.5)	209 (74.6)
Mild (%)	44 (16.7)	47 (17.9)	52 (19.8)	56 (22.0)	54 (20.0)	43 (15.6)	52 (19.3)	62 (22.1)
Moderate (%)	2 (0.8)	12 (4.6)	7 (2.7)	11 (4.3)	5 (1.9)	4 (1.4)	6 (2.2)	8 (1.9)
Malignant (%)	0 (0.0)	2 (0.8)	0 (0.0)	3 (1.2)	0 (0.0)	1 (0.4)	0 (0.0)	1 (0.4)

^∗^ *P* < 0.05 compared to quartile 1; ^¶^*P* < 0.05 compared to quartile 2. UACR: albumin/creatinine ratios; BMI: body mass index; BP: blood pressure; N/L: neutrophil to lymphocyte ratio; HDL-c: high-density lipoprotein cholesterol; LDL-c: low-density lipoprotein cholesterol; eGFR: estimated glomerular filtration rate.

**Table 3:** Characteristics and Mitchell–Wong classification stratified by sex.

	Male (*n* = 1044)	Female (*n* = 1096)	*P* value
Age (years)	71.8 ± 5.5	71.3 ± 5.5	0.139
BMI (kg/m^2^)	21.9 ± 3.2	21.9 ± 3.1	0.915
Systolic BP (mmHg)	136.7 ± 17.4	139.0 ± 17.5	0.031
Diastolic BP (mmHg)	79.3 ± 10.6	79.2 ± 10.4	0.884
N/L ratio	1.77 ± 0.89	1.77 ± 0.73	0.992
Fasting blood glucose (mg/dL)	98.4 ± 17.0	104.6 ± 16.1	<0.001
Cholesterol (mg/dL)	202.5 ± 37.1	206.3 ± 38.5	0.105
Triglycerides (mg/dL)	132.6 ± 98.9	138.9 ± 77.6	0.252
HDL-c (mg/dL)	61.0 ± 13.7	64.6 ± 14.7^∗^	<0.001
LDL-c (mg/dL)	113.8 ± 30.1	112.6 ± 29.9	0.937
eGFR (mL/min/1.73 m^2^)	89.8 ± 30.1	86.8 ± 29.9	0.027
UACR (mg/g)	5.70 ± 2.95	14.64 ± 2.60	<0.001
Albuminuria (%)	319 (30.6)	348 (31.8)	0.575
Mitchell–Wong classification			
None (%)	808 (77.4)	860 (78.5)	0.556
Mild (%)	199 (19.1)	211 (19.3)	0.913
Moderate (%)	32 (3.1)	23 (2.1)	0.173
Malignant (%)	5 (0.5)	2 (0.2)	0.363

UACR: albumin/creatinine ratios; BMI: body mass index; BP: blood pressure; N/L: neutrophil to lymphocyte ratio; HDL-c: high-density lipoprotein cholesterol; LDL-c: low-density lipoprotein cholesterol; eGFR: estimated glomerular filtration rate. Female patients had higher systolic BP, fasting blood glucose, HDL-c, and UACR but lower eGFR compared to male patients.

**Table 4:** Adjusted odds ratio for hypertension retinopathy by quartiles of UACR.

	Model 1	*P*	Model 2	*P*	Model 3	*P*
	OR (95%)		OR (95%)		OR (95%)	
Cohort (*n* = 2140)						
Quartile 1	1.0 (reference)		1.0 (reference)		1.0 (reference)	
Quartile 2	1.04 (0.78-1.40)	0.807	1.04 (0.77-1.40)	0.807	1.06 (0.78-1.44)	0.700
Quartile 3	1.15 (0.86-1.55)	0.357	1.15 (0.86-1.55)	0.357	1.20 (0.89-1.63)	0.309
Quartile 4	1.46 (1.10-1.95)	0.010	1.46 (1.10-1.95)	0.010	1.42 (1.05-1.92)	0.025
*P* for trends	<0.001		<0.001		<0.001	

Model 1: unadjusted. Model 2: adjusted for age and sex. Model 3: model 2 adjusted for BMI, systolic BP, diastolic BP, N/L ratio, fasting blood glucose, cholesterol, triglycerides, HDL-c, LDL-c, and eGFR. UACR: albumin/creatinine ratios; BMI: body mass index; BP: blood pressure; N/L: neutrophil to lymphocyte ratio; HDL-c: high-density lipoprotein cholesterol; LDL-c: low-density lipoprotein cholesterol; eGFR: estimated glomerular filtration rate; OR: odds ratio; CI: confidence index.

**Table 5:** Adjusted odds ratio for hypertension retinopathy by quartiles of UACR and by sex.

	Model 1	*P*	Model 2	*P*	Model 3	*P*
	OR (95%)		OR (95%)		OR (95%)	
Male (*n* = 1044)						
Quartile 1	1.0 (reference)		1.0 (reference)		1.0 (reference)	
Quartile 2	1.43 (0.94-2.21)	0.096	1.43 (0.94-2.21)	0.096	1.39 (0.90-2.15)	0.136
Quartile 3	1.37 (0.89-2.11)	0.121	1.37 (0.89-2.11)	0.121	1.27 (0.82-1.98)	0.290
Quartile 4	1.79 (1.18-2.73)	0.006	1.79 (1.18-2.73)	0.006	1.65 (1.07-2.55)	0.024
*P* for trends	<0.001		<0.001		<0.001	

Female (*n* = 1096)						
Quartile 1	1.33 (0.87-2.03)	0.190	1.33 (0.87-2.03)	0.190	1.40 (0.91-2.16)	0.127
Quartile 2	1.0 (reference)		1.0 (reference)		1.0 (reference)	
Quartile 3	1.30 (0.85-1.99)	0.228	1.30 (0.85-1.99)	0.228	1.34 (0.87-2.07)	0.1.77
Quartile 4	1.61 (1.07-2.44)	0.023	1.61 (1.07-2.44)	0.023	1.61 (1.06-2.45)	0.025
*P* for trends	<0.001		<0.001		<0.001	

Model 1: unadjusted. Model 2: adjusted for age and sex. Model 3: model 2 adjusted for BMI, systolic BP, diastolic BP, N/L ratio, fasting blood glucose, cholesterol, triglycerides, HDL-c, LDL-c, and eGFR. UACR: albumin/creatinine ratios; BMI: body mass index; BP: blood pressure; N/L: neutrophil to lymphocyte ratio; HDL-c: high-density lipoprotein cholesterol; LDL-c: low-density lipoprotein cholesterol; eGFR: estimated glomerular filtration rate; OR: odds ratio; CI: confidence index.

## Data Availability

Readers can access the data underlying the findings of the study by contacting the corresponding author.
